# Intelligent Control of Agricultural Irrigation through Water Demand Prediction Based on Artificial Neural Network

This article has been retracted.

**DOI:** 10.1155/2021/7414949

**Published:** 2021-11-23

**Authors:** Qiuyu Bo, Wuqun Cheng

**Affiliations:** Institute of Urban and Rural Construction, Agricultural University of Hebei, Baoding 071001, China

## Abstract

In irrigated areas, the intelligent management and scientific decision-making of agricultural irrigation are premised on the accurate estimation of the ecological water demand for different crops under different spatiotemporal conditions. However, the existing estimation methods are blind, slow, or inaccurate, compared with the index values of the water demand collected in real time from irrigated areas. To solve the problem, this paper innovatively introduces the spatiotemporal features of ecological water demand to the forecast of future water demand by integrating an artificial neural network (ANN) for water demand prediction with the prediction indices of water demand. Firstly, the ecological water demand for agricultural irrigation of crops was calculated, and a radial basis function neural network (RBFNN) was constructed for predicting the water demand of agricultural irrigation. On this basis, an intelligent control strategy was presented for agricultural irrigation based on water demand prediction. The structure of the intelligent control system was fully clarified, and the main program was designed in detail. The proposed model was proved effective through experiments.

## 1. Introduction

As a big agricultural country, China faces a severe shortage of agricultural irrigation water, owing to the low per-capita water resources and the imbalance between water supply and demand [1, 2]. Modern agriculture aims to achieve a high yield of high-quality crops in an ideal cycle. To promote agricultural development in China, it is very meaningful to reconstruct the irrigation water facilities in large irrigated areas, trying to detect an agricultural situation in real time, make reasonable plans for irrigation water consumption, and realize automatic water supply [3–5]. In irrigated areas, the intelligent management and scientific decision-making of agricultural irrigation is premised on the accurate estimation of the ecological water demand for different crops under different spatiotemporal conditions [6–8].

After analyzing the water supply and consumption features in local irrigated areas, Sun et al. [9] adjusted the weights of the indices in the current water consumption evaluation system through analytic hierarchy process (AHP) and constructed a time series prediction model to forecast the available water resources, industrial water demand, domestic water demand, and agricultural water demand in the irrigated areas with different assurance rates, thereby balancing the water supply with water demand in these areas. Essaid and Caldwell [10] numerically simulated the irrigation water demand of sweet potatoes and peanuts, predicted the accurate water-saving potential of irrigated areas, and put forward an adjustment strategy of the irrigation system to improve the water utilization rate.

To make full use of irrigation water, most irrigated areas choose to renovate the traditional irrigation management mode based on high-resolution remote sensing images. The water demand of irrigated areas is usually inverted and predicted through accurate detection of block changes [11, 12]. Nejatijahromi et al. [13] established a deep semantic segmentation network to classify the planting areas of different types of crops and introduced multiple indices to image fusion during the preprocessing of remote sensing images. In this way, the spectral complexity and spatial resolution were improved, and the feature information of irrigated area images was enhanced. Pani and Mishra [14] replaced the ordinary convolution and rectified linear unit (ReLU) of the U-Net semantic segmentation network with depthwise separable convolution and Mish activation function, respectively, thereby improving the classification accuracy of the planting areas of different crops. In addition, they constructed an inversion model for the water content in the soil at different depths, which couples the normalized difference vegetation index (NDVI) and automatic water extraction index. Foglia et al. [15] set up a dynamic multifactor prediction model for soil water content. Based on long short-term memory (LSTM) neural network, their model boasts a high prediction accuracy and a low degree of discretization. To predict water demand more accurately, Hassani and Shahdany [16] improved the multiplication of the Jacobian matrix in the Levenberg–Marquardt (LM) algorithm: this operation was replaced with gradient vector calculation and quasi-Hessian matrix. The improved LM algorithm was used as the learning algorithm for the fuzzy neural network of water demand prediction. The results show that the improved algorithm brings higher network learning efficiency and occupies a small storage space. Mimicking the information transmission mode of the cerebral cortex, Li et al. [17] designed a peaking mechanism for the structural growth and pruning of neural network and implemented it to predict the short-term water demand.

To a certain extent, the traditional estimation methods for the water demand in irrigated areas, namely, empirical formulas, hydrological methods, and microclimate methods, are blind and slow. Infrared remote sensing techniques can diagnose the water level by the physiological properties of crops, providing support to decision-makers in water development and management. However, these techniques are not accurate enough. To solve this problem, this paper combines an ANN for water demand prediction with the prediction indices of water demand.  Section 2 computes the ecological water demand for nonfixed crops in the agricultural irrigated area, using the simple and direct area quota method.  Section 3 predicts the water demand of crops in the agricultural irrigated area by integrating the radial basis function neural network (RBFNN) with autoregression model.  Section 4 presents an intelligent control strategy for agricultural irrigation based on water demand prediction and constructs a precision agricultural irrigation intelligent control system, which encompasses a distributed wireless sensor subsystem, a water demand prediction subsystem, and an agricultural irrigation control subsystem. The proposed model was proved effective through experiments.

## 2. Calculation of Ecological Water Demand

The water demand for agricultural irrigation refers to the amount of irrigation water that must be consumed to maintain the normal growth of crops. Given the uneven distribution of population and farmland in China, the planting area of water-demanding regular rice varieties is growing, and the homogeneity of crops is on the rise. To optimize water allocation and realize intelligent control of agricultural irrigation, it is important to scientifically calculate and accurately predict water demand indices of agricultural irrigation.

Firstly, this paper uses the relatively simple and direct area quota method to compute the irrigation water demand of an irrigated area: multiply the size of the irrigated area with the ecological water demand quota of each crop and superimpose the products. Let *ZS* be the total water demand of the irrigated area and *ZS*_*i*_, *P*_*i*_, and *Q*_*i*_ the ecological water demand, planting area, and ecological water demand quota of crop *i*, respectively. Among them, the quota can be obtained through experimental analysis and theoretical calculation. Assuming that there are *m* crops, then *ZS* can be calculated by

(1) $$\begin{array}{c} ZS=\sum_{i=1}^{m}ZS_{i}=\sum_{i=1}^{m}P_{i}\cdot Q_{i}. \end{array}$$

In arid areas, crop growth mainly relies on groundwater and irrigation. This paper directly estimates the actual ecological water demand of crops in arid and semiarid areas, using phreatic water evaporation, which requires only a few parameters. Let *WZS* be the total ecological water demand of vegetation; *ZS*_*ij*_ and *DV*_*ij*_ the ecological water demand and phreatic water evaporation of crop *i* in month *j*, respectively; and Ψ_*V*_ the vegetation index of crops. Then, *ZS* can be calculated by

(2) $$\begin{array}{c} ZS=\sum_{i=1,j=1}^{m}ZS_{ij}=\sum_{i=1,j=1}^{m}P_{i}\cdot DV_{ij}\cdot \Psi_{V}. \end{array}$$

Let *e*_1_ and *e*_2_ be empirically coefficients; *DB*_*i*_ the buried depth of groundwater at the location of crop *i*; *DB*_max_ the ultimate buried depth for phreatic water evaporation; and *DV*_*j*_^*θ*^ the surface evaporation of regular evaporation dish in month *j*. Then, *DV*_*ij*_ can be calculated by Aver'yanov's phreatic evaporation formula:

(3) $$\begin{array}{c} DV_{ij}=e_{1}{\left(\frac{1-DB_{i}}{DB_{\max}}\right)}^{e_{2}}DV_{j}^{\theta }. \end{array}$$

During crop growth, transpiration consumes the largest amount of water. In this paper, the actual evapotranspiration is used to determine the ecological water demand of each crop. The calculation assumes that the water supply is sufficient. Let *DV*_*j*_^*∗*^ be the evapotranspiration caused by the transpiration of the reference crop in month *j* and Ψ_*T*_ the soil moisture correction coefficient of the irrigated area. Then, the maximum ecological water demand of a crop can be calculated by

(4) $$\begin{array}{c} ZS=\sum_{i=1,j=1}^{m}ZS_{ij}=\sum_{i=1,j=1}^{m}P_{i}\cdot DV_{ij}, \end{array}$$

where *DV*_*ij*_ can be calculated by

(5) $$\begin{array}{c} DV_{ij}=DV_{j}^{*}\times \Psi_{V}\times \Psi_{T}. \end{array}$$

The Penman–Monteith equation, recommended by The United Nations Food and Agriculture Organization (FAO), was adopted to compute the potential evaporation *DV*^*∗*^ of crops in an irrigated area. Let Γ be the slope between the temperature change curve and the saturated vapor pressure; *FS* the net radiation of crop surface; *TH* the heat flux of the soil in the irrigated area; *δ* the psychrometer constant; *T*_*AV*_ the mean temperature; *v*_*f*_ the wind speed at a fixed height; and *AV*_*B*_ and *AV*_*R*_ saturated and actual vapor pressures, respectively. Then, *DV*^*∗*^ can be calculated by

(6) $$\begin{array}{c} DV^{*}=\frac{0.4\Gamma \left(FS-TH\right)+\delta \left(900/\left(T_{AV}+273\right)\right)v_{f}\left(AV_{B}-AV_{R}\right)}{\Gamma +\delta \left(1+0.35v_{2}\right)}. \end{array}$$

The slope Γ can be calculated by

(7) $$\begin{array}{c} \Gamma =\frac{4100\times 0.62\left(17.3T_{AV}/\left(T_{AV}+327.3\right)\right)}{{\left(T_{AV}+327.3\right)}^{2}}. \end{array}$$

The net radiation of crop surface *FS* is the difference between net short-wave radiation *FS*_*D*_ and net long-wave radiation *FS*_*C*_:

(8) $$\begin{array}{c} FS=FS_{D}-FS_{C}. \end{array}$$

Let *FS*_*S*_ be solar radiation; *m*_*S*_ the actual sunshine hours; and *M*_*S*_ the most probable sunshine hours. Then, *FS*_*D*_ can be calculated by

(9) $$\begin{array}{c} FS_{D}=0.78\left(\frac{1}{4}+\frac{m_{s}}{2M_{S}}\right)FS_{S}. \end{array}$$

Let Φ_*S*_ be the solar constant; *θ* the latitude; and *DO* the day order. Then, solar radiation *FS*_*S*_ can be calculated by

(10) $$\begin{array}{c} FS_{S}=\frac{24\times 60}{\pi }\times \Phi_{S}\times RDR_{SE}\left[HA_{S}\sin\;\theta \;\;\sin\;\gamma +\cos\;\theta \;\;\cos\;\gamma HA_{S}\right]. \end{array}$$

The reciprocal *RDR*_*SE*_ of the relative distance between the Sun and the Earth can be calculated by

(11) $$\begin{array}{c} RDR_{SE}=1+\frac{1}{30}\cos\left(\frac{2\pi }{365}\times DO\right). \end{array}$$

The solar hour angle *HA*_*S*_ in formula (10) can be calculated by

(12) $$\begin{array}{c} HA_{S}=ar\;\cos\left[-\tan\;\theta \;\tan\;\gamma \right]. \end{array}$$

The solar magnetic declination *γ* in formula (10) can be calculated by

(13) $$\begin{array}{c} \gamma =0.4\;\sin\left(\frac{2\pi }{365}DO-1.4\right). \end{array}$$

Let *MT*_max-*j*_ and *MT*_min-*j*_ be the maximum and minimum absolute temperatures of month *j*. Then, the net long-wave radiation *FS*_*C*_ can be calculated by

(14) $$\begin{array}{c} FS_{C}=4.903\times 10^{-9}\left(1.35\frac{0.25+0.5\left(m_{S}/M_{S}\right)}{0.75+2\times \left(c/100000\right)}-0.35\right)\left(0.34-0.14\sqrt{AV_{R}}\right)\left(\frac{{\left(MT_{\max-j}\right)}^{4}+{\left(MT_{\min-j}\right)}^{4}}{2}\right). \end{array}$$

Let *DT*_max-*k*_ and *DT*_min-*k*_ be the daily mean maximum and minimum temperatures of day *k*; *SD*_*AV*_ the daily mean relative humidity; and *v*_*c*_ the wind speed at the altitude of *c* meters. Then, the saturated vapor pressure *AV*_*B*_ can be calculated by

(15) $$\begin{array}{c} AV_{B}=\frac{r\left(DT_{\max-k}\right)+r\left(DT_{\min-k}\right)}{2}, \end{array}$$

where *r* is exponentiation:

(16) $$\begin{array}{c} r\left(t\right)=0.62e^{17.28t/\left(t+327.3\right)}. \end{array}$$

The actual vapor pressure *AV*_*R*_ can be calculated by

(17) $$\begin{array}{c} AV_{R}=\frac{AV_{B}\times SD_{AV}}{100}. \end{array}$$

Suppose the height is fixed at 2 m. Then, the mean wind speed can be calculated by

(18) $$\begin{array}{c} v_{f}=v_{c}\frac{4.9}{\ln\left(67.8c-5.4\right)}. \end{array}$$

## 3. RBFNN-Based Water Demand Prediction

### 3.1. Network Construction

To predict the crop water demand in the agricultural irrigated area, this paper sets up a prediction model based on RBFNN, which boasts a strong approximation ability and a fast convergence speed. As shown in Figure 1, the RBFNN consists of three layers: an input layer that connects and transmits external signals, a hidden layer that realizes RBF mapping, and an output layer that performs linear summation. The input layer receives the sample data about the parameters required to compute the crop water demand in the target irrigated area. The RBF mapping, which underpins the nonlinear transform between the input layer and hidden layer, constitutes the basis of the hidden layer. Therefore, the output of the RBFNN can be regarded as a linear combination of basis functions derived from hidden layer nodes.

The RBF centers were solved through clustering. Let *B*: ℝ^*K*^ ⟶ ℝ^*O*^ be the mapping response of RBF; *a*_*i*_ the data of index sample *i* imported to the input layer, that is, the real-time data series of water demand indices for agricultural irrigation; *A = *(*a*_l_, *a*_2_,…)^*T*^* *∈* *ℝ^*K*^ the input vector; *b*_*k*_ the output of output layer node *k*; *ω*_*k*_ the connection weight between all hidden layer nodes and output layer node *l*; *W*_*G*_ the center *G* of hidden layer nodes; *J* and *K* the number of hidden layer centers and the total number of input layer nodes; *F*(∙) the basis function; and ‖·‖ the Euclidean norm. Then, the RBFNN output can be expressed as

(19) $$\begin{array}{c} b_{k}=\sum_{i=1}^{K}\sum_{G=1}^{J}\omega_{i}\left(i,H\right)F\left({\left\|a_{i}-W_{G}\right\|}^{2}\right). \end{array}$$

The hidden layer output based on Gaussian function can be calculated by

(20) $$\begin{array}{c} c_{l}=\theta \left(\sum_{i=1}^{K}\sum_{G=1}^{J}\frac{{\left(a_{i}-W_{G}\right)}^{2}}{\gamma_{G}^{2}}\right). \end{array}$$

To sum up, RBFNN has three adjustable parameters: variance, center position, and output layer weight. Under the premise that training index samples can reflect the essence of crop water demand prediction in the irrigated area, *n*_*W*_ uniformly distributed centers were selected with an interval of *q*, that is, network centers. On this basis, the variance *s* = *q*/(2*n*_*W*_)^−2^ of the Gaussian function can be solved.

### 3.2. Determination of Network Parameters

The RBF centers were determined through fuzzy *k* means (FKM) clustering of unsupervised self-organizational learning. Let *A*_*US*_ *=* (*A*_l_, *A*_2_,…, *A*_*N*_) be the set of *N* index samples imported for unsupervised learning; *U* the number of clusters; *D* *=* [*d*_*il*_]_*U×N*_ the membership matrix of sample *l* in cluster *i*; *d*_*il*_ the membership function of sample *l* in cluster *i*; *O* *=* [*o*_1_, *o*_2_,…, *o*_*U*_] the set of cluster centers; *ξ*_*il*_ the distance from *a*_*l*_ to *o*_*i*_; *ε* the weighted index of the network; and *σ* the allowable error. To minimize the weighted sum of squares of the distance between sample center and cluster centers, an objective function of classification *J*(*D*, *O*) = ∑_*l*=1_^*N*^∑_*i*=1_^*U*^(*d*_*il*_)^*N*^(*ξ*_*il*_^2^) can be constructed and minimized. The detailed operations go as follows:

Step 1: initialize the network, set the initial number of iterations *t* = 0, and determine the initial values of *N*, *U*, and *D*^(*t*)^.
Step 2: derive the following from *D*^(*t*)^:
  (21) $$\begin{array}{c} o_{i}=\frac{1}{\sum_{l=1}^{N}{\left(d_{il}\right)}^{\varepsilon }}\sum_{l=1}^{\varepsilon }{\left(d_{il}\right)}^{N}a_{il},\;i=1,2,\ldots ,U. \end{array}$$
Step 3: suppose *l* = 1,…, *N.* The set of clusters satisfying the condition that the distance between sample center and cluster center is zero can be expressed as
  (22) $$\begin{array}{c} Q_{l}=\left\{i|0\leq i\leq U,\xi_{il}=\left\|a_{l}-o_{i}\right\|=0\right\}. \end{array}$$
The set of the other clusters can be described by
  (23) $$\begin{array}{c} Q^{*}=\left\{1,2,\ldots ,U\right\}-Q_{l}. \end{array}$$
If *Q*_*l*_ is an empty set, then
  (24) $$\begin{array}{c} d_{il}=\frac{1}{\sum_{j=1}^{U}{\left(\xi_{il}/\xi_{jl}\right)}^{2/\left(\varepsilon -1\right)}}. \end{array}$$
If *Q*_*l*_ is not an empty set, then *d*_*il*_ = 0, *i* belongs to set *Q*_*l*_, and Σ_*i*∈*Il*_*d*_*il*_ = 1. Make *l* = *l* + 1, and return to the start of Step 3.
Step 4: if ‖*D*^(*t*)^ − *D*^(*t*+1)^‖ is smaller than the learning convergence rate *η*, then terminate the network training. If ‖*D*^(*t*)^ − *D*^(*t*+1)^‖ is greater than *η*, add one to the number of iterations and return to the start of Step 2.

The hidden node width of RBFNN was determined by the k-nearest neighbors (KNN) algorithm. First, the sum of the distances from a sample center to the centers of the nearest *K* clusters was averaged. Then, the width was derived from the mean value. Let *o*_*j*_′ be the sample center closest to cluster center *o*_*i*_. Then, the width of hidden layer nodes can be expressed as

(25) $$\begin{array}{c} HW_{i}=\frac{1}{l}\sum_{j=1}^{l}\left\|o_{i}-o_{j}^{\prime }\right\|. \end{array}$$

Let Gauss(*a*) be the Gaussian function. Then, the RBF can be approximated by the following function:

(26) $$\begin{array}{c} AF\left(a\right)=\sum_{i=1}^{U}\omega_{i}\times \text{Gauss}\left(\left\|a-o_{i}\right\|\right). \end{array}$$

Solving the approximation function is equivalent to minimizing the following cost function by adjusting the weight set {*ω*_*i*_*|i* *=* 1, 2,…, *U*}:

(27) $$\begin{array}{c} \Phi \left(AF^{*}\right)=\sum_{l=1}^{N}{\left[\xi_{l}-AF\left(a_{l}\right)\right]}^{2}+\mu {\left\|NOR^{*}\right\|}^{2}=\sum_{l=1}^{N}{\left[\xi_{l}-\sum_{i=1}^{g}\omega_{i}\text{Gauss}\left(\left\|a_{l}-o_{i}\right\|\right)\right]}^{2}+\mu {\left\|NOR^{*}\right\|}^{2}, \end{array}$$

where the first term is the standard error and the second term is the regularization term to satisfy the requirements on continuity and smoothness. Formula (27) can be sorted out as

(28) $$\begin{array}{c} \Phi \left(U^{*}\right)=\sum_{l=1}^{N}{\left[\xi_{l}-\text{Gauss}\cdot \omega \right]}^{2}+\mu {\left({\text{NOR}}^{*},{\text{NOR}}^{*}\right)}_{{}^{M}}^{2}={\left\|\xi_{l}-\text{Gauss}\cdot \omega \right\|}^{2}+\mu \omega^{T}H_{0}\omega , \end{array}$$

where

(29) $$\begin{array}{c} \xi ={\left(\xi_{1},\xi_{2},\ldots ,\xi_{N}\right)}^{T};\\ \omega ={\left(\omega_{1},\omega_{2},\ldots ,\omega_{U}\right)}^{T},\\ \text{Gauss}=\left[\begin{array}{cccc} g\left(a_{1},o_{1}\right) & g\left(a_{1},o_{2}\right) & \ldots & g\left(a_{1},o_{U}\right)\\ g\left(a_{2},o_{1}\right) & g\left(a_{2},o_{2}\right) & \ldots & g\left(a_{2},o_{U}\right)\\ \vdots & \vdots & \ldots & \vdots \\ g\left(a_{N},o_{1}\right) & g\left(a_{N},o_{2}\right) & \ldots & g\left(a_{N},o_{U}\right) \end{array}\right]. \end{array}$$

Minimizing Φ(*AF*^*∗*^),

(30) $$\begin{array}{c} \left(g^{T}g+\mu g_{0}\right)\omega =g^{T}\xi . \end{array}$$

The solution of the RBF approximation function should be normalized by

(31) $$\begin{array}{c} \omega ={\left(g^{T}g+\mu g_{0}\right)}^{-1}g^{T}\xi . \end{array}$$

After setting *l* = *l* + 1, the network iteration can be described by

(32) $$\begin{array}{c} \omega_{l+1}=\omega_{l}-\chi \frac{\gamma \Phi \left(U\right)}{\gamma \omega_{k}}=\omega_{l}-\chi \left[\left(g^{T}g+\mu g_{0}\right)\omega_{l}-g^{T}\xi \right]. \end{array}$$

### 3.3. Construction of Hybrid Prediction Model

For accurate prediction of the water demand of agricultural irrigation, this paper combines RBFNN with an autoregression model into a water demand prediction model. In the model, the coefficient of the autoregression function can be approximated by the RBFNN.

Let *u*_*b*_ be the order of the model; *O*_*l*_^*i*^ the center of RBFNN index samples; *μ*_*l*_ the scale ratio; *υ*_0_ and *υ*_*bi*_ the state coefficients of the model; *s*_*l*_^0^ and *s*_*il*_^*s*^ the vector constants of the model; *A*(*t* − 1) the index sample determining the output state of the time-varying model; and *NO*(*t*) the white noise. Then, the proposed prediction model can be established as

(33) $$\begin{array}{c} \left\{\begin{array}{c} b\left(t\right)=\upsilon_{0}\left(A\left(t-1\right)+\sum_{i=1}^{u_{b}}\upsilon_{bi}\left(A\left(t-1\right)\right)b\left(t-i\right)+NO\left(t\right)\right),\\ \upsilon_{0}\left(A\left(\tau -1\right)\right)=s_{0}^{0}+\sum_{l=1}^{N}e^{-\mu_{l}^{b}{\left\|A\left(\tau -1\right)-O_{l}^{b}\right\|}_{2}^{2}},\\ \upsilon_{bi}\left(A\left(\tau -1\right)\right)=s_{i0}^{b}+\sum_{l=1}^{N}s_{il}^{b}e^{-\mu_{l}^{b}{\left\|A\left(\tau -1\right)-O_{l}^{b}\right\|}_{2}^{2}},\\ O_{l}={\left(O_{l,1},O_{l,2},\ldots ,O_{l,N}\right)}^{T}. \end{array}\right. \end{array}$$

The weighted prediction result obtained from the water demand indices in Section 2 was combined with the prediction result of the RBFNN in Section 3, using validity weights.  Figure 2 explains the steps of our hybrid prediction model. Firstly, the real-time data series of water demand indices for agricultural irrigation was divided into a training set and a test set. The two sets were used separately to predict the water demand. Then, the predicted water demand was compared with the actual water demand of the agricultural irrigated area. The error between them was reduced to realize intelligent control of agricultural irrigation. Then, the validity weights *ω*′ and *ω*″ of the two methods were calculated.

The core of the intelligent control system for agricultural irrigation is a single-chip microcomputer (SCM) connected to a triode amplifier circuit, which drives a relay. The opening/closing of the solenoid valve is controlled by the contact of the relay. Because of the small power of the selected solenoid valve, the triode type being adopted can stabilize the voltage and current and ensure the reliable functioning of the system. The soil humidity sensor transmits the humidity to the irrigation monitoring control system. The read humidity is compared with the preset lower bound of humidity to control the level at the pins of the SCM, in order to execute the irrigation mode.

During the intelligent control of actual agricultural irrigation, *ω*′ and *ω*″ change with the updates of the control signals of the irrigation solenoid valve, in order to improve the precision of irrigation control.

Similarly, the test set was predicted separately by two methods. Then, the final hybrid prediction result was obtained through the weighted calculation, using the validity weights *ω*′ and *ω*″. The final step is to evaluate the accuracy of water demand prediction.

## 4. Intelligent Control Strategy Based on Water Demand Prediction

Based on the hybrid prediction of water demand for agricultural irrigation, the authors developed a precision irrigation intelligent control system (Figure 3), which encompasses a distributed wireless sensor subsystem, a water demand prediction subsystem, and an agricultural irrigation control subsystem. The agricultural irrigation control subsystem evaluates whether the target crop needs water by comparing soil humidity with predicted crop water demand. If the crop needs water, the solenoid valve will be launched for irrigation. The duration of irrigation will be controlled by the water quota for agricultural irrigation.  Figure 4 shows the signal conversion in the distributed wireless sensor subsystem, which measures soil humidity in real time, and the agricultural irrigation control subsystem, which predicts the indices of crop water demand.

The analog signal from the wireless soil humidity sensor has a low voltage. After passing through the amplifier circuit, the voltage is increased to the useable level. Then, the analog signal is converted by the converter into a digital signal. After that, the SCM level is transformed by the chip into the level for the serial port of the host, which supports intelligent control.

The precision irrigation intelligent control system should operate rapidly while occupying a small memory. For this purpose, Keil *µ* Vision 4.0, which contains efficient C compilers and project managers, was selected to compile the program code of the system. The main program flow is presented in Figure 5. Once the intelligent control system starts, the main program will be initialized, and the command will be read. When the water demand surpasses the actual soil humidity, the solenoid valve will be opened to start sparkling irrigation in the irrigated area. The irrigation will last until the end of the preset duration. Then, the valve will be closed to terminate the irrigation.

## 5. Experiments and Results Analysis

In the agricultural irrigated area, the phreatic evaporation of crops is greatly affected by the actual atmospheric evaporation capacity.  Figure 6 presents the monthly mean evaporations of different planting zones in the agricultural irrigated area, which were derived from the daily observation data. It can be inferred that the crop evaporation was relatively large from June to September. The change trend meets the actual variation of water demand.

During the estimation of the ecological water demand of vegetation, the key of the area quota method lies in determining the ecological water demand quota of each type of plant. In the target irrigated area, the irrigation quotas for soybean and corn are 5,100 and 4,960 m^3^/hm, respectively. Considering the planting areas and expansion goals of the crops in the current year, the area quota method was employed to compute the ecological water demands of soybean and corn in the irrigated area. The results (Table 1) show that the current ecological water demand of soybean and corn in the target irrigated area was 1.856 and 4.182 m^3^, respectively. The total water demand reached 6.028 m^3^. Under the expansion goals, the ecological water demand of soybean and corn was predicted as 4.371 and 4.352 m^3^, respectively. The total water demand reached 8.723 m^3^. The traditional agricultural irrigation control systems are very inefficient in water use. The irrigation water utilization coefficient is as low as 0.6. Based on this coefficient, the actual ecological water demand of soybean and corn in the target irrigated area was 1.235 and 2.372 m^3^, respectively. The total water demand reached 3.607 m^3^. By contrast, our precision irrigation intelligent control system can elevate the utilization coefficient to 0.85. On this basis, the actual ecological water demand of soybean and corn in the target irrigated area was 3.464 and 3.375 m^3^, respectively. The total water demand reached 6.839 m^3^.

By the phreatic evaporation method, the ecological water demand of crops per unit area in the target irrigated area averaged at 2,749 m^3^/hm. The predicted values under the expansion goals are given in Table 2. It can be seen that the total annual ecological water demand of soybean in the irrigated area was 2.322 m^3^, and that of corn was 2.573 m^3^. The total water demand reached 4.895 m^3^.

By the vegetation evapotranspiration method, the mean ecological water demand of crops per unit area in the target irrigated area was 3,359 m^3^/hm. The predicted values under the expansion goals are given in Table 3. It can be seen that the total annual ecological water demand of soybean in the irrigated area was 2.841 m^3^, and that of corn was 2.597 m^3^. The total water demand reached 5.438 m^3^.

Figures 7 and 8 compare the predicted water demands for the target irrigated area and prediction errors, respectively.  Table 4 sums up the absolute errors of water demand prediction by different methods. The error metrics include maximum absolute error, mean absolute error, and root mean square of absolute error. From Figures 7 and 8 and Table 4, it can be inferred that the chaotic model, traditional RBF model, and our hybrid prediction model all achieved high accuracy in forecasting the water demand in the irrigated area. However, the three error metrics of our model were way smaller than those of other models. Therefore, our method can adapt well to the index value fluctuations in prediction and realize stable prediction performance, compared with the chaotic model and traditional RBF model.

## 6. Conclusions

This paper presents an intelligent control method for agricultural irrigation through ANN-based water demand prediction. Firstly, the ecological water demand for agricultural irrigation of crops was calculated, and an RBFNN was constructed for predicting the water demand of agricultural irrigation. Then, the authors developed an intelligent control strategy for agricultural irrigation based on water demand prediction, detailed the structure of the intelligent control system, and designed the main program. Through experiments, the ecological water demand for crops in the targeted irrigated area was separately calculated by the area quota method, the phreatic evaporation method, and the vegetation evapotranspiration method, providing the data support to the weighted prediction of water demand indices. Then, the authors compared the predicted water demands for the target irrigated area and prediction errors, respectively, and demonstrated that our method could predict the water demand in the irrigated area more accurately and stably than other models.

This paper preliminarily explores and discusses the calculation of agricultural irrigation water demand. There are several limitations of the work, which need to be improved in the future. (1) Due to data availability, the meteorological data are the mean of the three stations around the study area. Thus, the calculated evaporation may deviate from the actual evaporation in the study area. (2) The correlation between groundwater level and vegetation area is not fully demonstrated. The vegetation response to groundwater level needs to be deeply analyzed in the future.

## Figures and Tables

**Figure 1:** Structure of RBFNN.

**Figure 2:** Steps of our hybrid prediction model.

**Figure 3:** Structure of intelligent control system.

**Figure 4:** Signal conversion in subsystems.

**Figure 5:** Main program flow.

**Figure 6:** Monthly mean evaporations of different zones in an irrigated area.

**Figure 7:** Comparison of predicted water demands.

**Figure 8:** Comparison of prediction errors.

**Table 1:** Ecological water demand obtained by area quota method.

Crop	Irrigation quota	Current state			Predicted state		
		Area	Calculated water demand	Actual water demand	Area	Calculated water demand	Actual water demand
Soybean	5,100	35,712	1.856	1.235	78,512	4.371	3.464
Corn	4,960	89,643	4.182	2.372	93,256	4.325	3.375

**Table 2:** Ecological water demand obtained by the phreatic evaporation method.

Crop	Ecological water demand						
	January	February	March	April	May	June	Full year
Soybean	0.023	0.051	0.139	0.278	0.356	0.368	2.322
Corn	0.027	0.056	0.161	0.306	0.375	0.409	2.573
	July	August	September	October	November	December	
Soybean	0.351	0.306	0.224	0.152	0.051	0.023	
Corn	0.401	0.358	0.246	0.143	0.069	0.022	

**Table 3:** Ecological water demand obtained by vegetation evapotranspiration method.

Crop	Ecological water demand						
	January	February	March	April	May	June	Full year
Soybean	0.012	0.023	0.065	0.113	0.518	0.532	2.814
Corn	0.021	0.053	0.168	0.305	0.358	0.409	2.597
	July	August	September	October	November	December	
Soybean	0.560	0.473	0.251	0.182	0.062	0.023	
Corn	0.401	0.358	0.260	0.153	0.076	0.035	

**Table 4:** Absolute errors of water demand prediction.

	Method	Maximum	Mean	Root mean square
Water demand prediction	Chaotic method	0.3	0.115	0.1235
	RBFNN	0.15	0.0965	0.1053
	Our hybrid prediction method	0.13	0.028	0.0342

## Data Availability

The data used to support the findings of this study are available from the corresponding author upon request.
